# Biochemical profile of milk thistle (*Silybum Marianum* L.) with special reference to silymarin content

This article has been retracted.

**DOI:** 10.1002/fsn3.1990

**Published:** 2020-11-09

**Authors:** Maryam Aziz, Farhan Saeed, Nazir Ahmad, Aftab Ahmad, Muhammad Afzaal, Shahzad Hussain, Abdellatif A. Mohamed, Mohamed S. Alamri, Faqir Muhammad Anjum

**Affiliations:** ^1^ Department of Food Sciences Government College University Faisalabad Pakistan; ^2^ Department of Food Science & Nutrition King Saud University Riyadh Saudi Arabia; ^3^ University of The Gambia Sere Kunda Gambia

**Keywords:** Chemical, Milk Thistle, Nutrition, Silymarin

## Abstract

The main objective of current study was to evaluate the antioxidant potential and nutritional composition of milk thistle with special reference to silymarin. For the purpose, different varieties of milk thistle were procured from three different cities of Pakistan. The study was comprised of three different phases. In 1st phase, nutritional composition, that is, moisture, fat, protein, fiber, and nitrogen free extract, was determined according to their respective methods. Moreover, antioxidant potential and quantification of silymarin content were explored in 2nd phase. Furthermore, in last phase, milk thistle seeds tea was developed and evaluated for nutritional and sensorial characteristics. At last, data obtained from each parameter was subjected to appropriate statistical design to determine the level of significance. Results showed significant difference in the nutritional and chemical composition of different milk thistle varieties as well as locations. Moreover, moisture content, ash content, fat content, fiber content, protein content, and NFE varied from 6.27% to 5.01%, 2.37 to 1.25%, 23.19 to 19.74%, 7.4 to 4.39%, 30.09 to 20.74%, and 45.42 to 34.13%, respectively. Furthermore, silymarin content quantified though HPLC ranged from 1669.5 mg/g to 1607.6 mg/g for soxhlet extract whereas, 1,840.6 mg/g to 1765.9 mg/g for microwave‐assisted extraction extract. Conclusively, it was depicted from the results that in case of variety, Blue was the best than White whereas, Islamabad was best in case of location.

## Graphical abstract

Milk thistle is safe, well tolerated in different preparation form and producing no any serious side effects. Milk thistle seeds can be used in raw form or made into a tea. Milk thistle seed tea has significant attention, both in scientific and consumer communities owing to its health benefits against variety of maladies. Furthermore, it is exposed that overall anti‐oxidant level improves in humans by using milk thistle tea. The free radicals quenching ability of milk thistle tea is better than black tea.

## 1 INTRODUCTION

Herbs fundamentally, plants or part of plants used for the treatment of many physiological disorders due to the presence of many phytochemicals and medicinal properties. Among these, milk thistle is an important herb playing a role as an antioxidant. This herb botanically known as *silybum marianum*, belongs to family, Asteraceae (Li et al., 2012). Milky white veins present on the leaves when broken their leaves these veins produce milky fluid due to this reason this herb named as milk thistle. Milk thistle have two types White and Blue (Evans, 2002; Rainone, 2005). Silybum marianum seeds comprises of oil content 26.05%, moisture content 4.48%, ash content 1.93%, crude fiber 5.48%, carbohydrates content 87.2% and total proteins 23% (Khan et al., 2007). The active constituents present in the seeds of the milk thistle are apigenin, silybonol, proteins, betaine, fixed oil, and free fatty acids (Marderosian, 2001).

The main bioactive component of medicinal plant (milk thistle) is silymarin. Silymarin is the mixture of different flavonolignans such as, silybinin A and B (SBN A&B), isosilybinin A and B (ISBN A&B), silychristin (SCN), and silydianin (SDN) (Anthony & Saleh, 2013; Li et al., 2008). It is a well‐known Chinese herb (Radek et al., 2007). Silymarin present in the seeds, fruit as well as in the leaves of the milk thistle but the seed part has the maximum concentration of silymarin (Hobbs, 2008). Silymarin content in the fruit of the milk thistle varies depend on the milk thistle varieties, geographic and climate changes in which it grows (Ghahreman, 1999). Milk thistle is used as medicine for the management of different diseases due to the presence of phytoconstituents such as antioxidants and total phenolics presence.

Milk thistle comprises high amount of oil due to this reason silymarin extraction is impossible in one step. Oil should be removed from the seeds before extraction of silymarin as it is the by‐product of silymarin industrial production. For recovery and purification of silymarin from silybum marianum plant seeds, extraction is first and important step. Studies described many different extraction methods for the extraction of silymarin from milk thistle plant seeds (Alvarez et al., 2003; Benthin et al., 1999; Wallace et al., 2003). Microwave‐assisted method, sample pretreatment, soxhlet extraction and reflux mercerization (With or without shaking) are the locally applied extraction methods (Mani et al., 2007). Now days, Microwave‐assisted extraction (MAE) has been usually documented as a useful, simple, and effective extraction method. When extraction is done through microwave than high extraction yield obtained in less time by using less solvent at same temperature (Hoang et al., 2007; Rohner et al., 2004; Teo et al., 2008; Zygmunt & Namiesnik, 2003; Huie, 2002).

Different preparations of milk thistle are safe and well tolerated with no any serious side effects. Commercially standardized extract of the milk thistle seeds are accessible in the form of tablets, tincture, extract, and capsule (Barceloux, 2008). Milk thistle seeds can be used in raw form or made into a tea (Bhattacharya, 2011). Milk thistle tea has antioxidant power due to the presence of flavonoid (silymarin) that treats liver issues and promote healthier liver functions. Moreover, reduces the bad LDL cholesterol level and total cholesterol level in the body.Tea decreases the nucleic acid, lipid membranes and proteins damage by trapping reactive oxygen species (ROS), for example, singlet oxygen, superoxide, proxy radicals, and hydroxyl. Furthermore, antioxidant level improves in humans by using milk thistle tea. The free radicals quenching ability of milk thistle tea is better than black tea.

## 2 MATERIALS AND METHODS

### 2.1 Procurement of raw materials

Milk thistle white and blue varieties were procured from three different cities (Islamabad, Faisalabad, Jhang) of Pakistan.

### 2.2 Proximate analysis

Proximate analysis of milk thistle was carried out for moisture content, crude protein, crude fat, crude fiber, ash, and NFE according to their respective methods as described in AACC (2000).

### 2.3 Extraction of silymarin

For this purpose, two extraction techniques soxhlet and microwave‐assisted extraction were employed for extraction of silymarin from milk thistle seeds.

### 2.4 Preparation of extract with soxhlet

A soxhlet apparatus, equipped with a 500 ml boiling flask, was used for extraction. 30 g of powder seeds were placed in a cellulose extraction thimble, 300 ml of n‐hexane was used as defatting solvent. Then this defatted powder was treated with 300 ml of solvent (methanol) for extraction. The extraction cycle started when the solvent began to boil and lasted for 6 hr. Extract were filter through Whatman filter paper and concentrated using rotary evaporation. Concentrates were stored in refrigerator for further analysis (Cagdas et al., 2011).

### 2.5 Preparation of extract with Microwave extraction

The powder seeds (5 g) and 95 ml solvent were treated in microwave oven specialized for extraction purpose. Firstly, seeds were defatted and then extract was prepared. Extract was filter through Whatman filter paper and concentrated using rotary evaporation. Concentration was stored in refrigerator for further analysis (Aslam et al., 2012).

### 2.6 Quantification of extracts with HPLC

HPLC analysis was performed on Shimadzu (Japan) HPLC instrument consisting of pump LC‐10AT, UV‐VIS detector 2SPD‐10AV. The analysis of silymarin samples were carried out by using C18 column. A mixture of phosphoric acid–methanol–water used as mobile phase. The elution was made in an isocratic mode at a flow‐rate 1 ml/min and the UV‐detector was used with wavelength at 288 nm. The quantitative analysis was based on silymarin standard and external standard method was used. Standard and sample were dissolved in the mobile phase for further processing (Radjabian et al., 2008 and Kvasnicka et al., 2003).

### 2.7 Antioxidant activity of milk thistle seeds extract

The antioxidant extract obtained from milk thistle seeds were analyzed for their antioxidant potential through different parameters like total phenolic content were measured by using Folin‐Ciocalteu method following the protocol of Singleton et al. (1999). Total phenolic content was estimated as gallic acid equivalent (mg gallic acid/g), total flavonoids content was estimated using the method of Ordon‐ez et al. (2006) free radical scavenging activity (DPPH assay) was measured using the protocol of Muller et al. (2011) and Vles and Gottenbos (1989) method was used to measure the reducing capacity of extracts.

### 2.8 Milk thistle tea

Tea was prepared from the milk thistle seeds. For the purpose MTS were roasted in hot air oven at temperature 210 for three different time intervals 20, 25, 30 min.

### 2.9 Antioxidant activity of milk thistle seeds tea

Tea obtained from milk thistle seeds were analyzed for their antioxidant potential through different parameters like total phenolic content were measured by using Folin‐Ciocalteu method following the protocol of Singleton et al. (1999). Total phenolic content was estimated as gallic acid equivalent (mg gallic acid/g) total flavonoids content were estimated using the method of Ordon‐ez et al. (2006) free radical scavenging activity (DPPH assay) was measured using the protocol of Muller et al. (2011) and Vles and Gottenbos (1989) method was used to measure the reducing capacity of tea.

### 2.10 Sensory evaluation

The milk thistle tea was subjected to sensory evaluation by trained taste panel using nine‐point hedonic scale system (9 = extremely; 1 = dislike extremely) as described by Meilgaard et al. (2007). Sensory evaluation regarded attributes like color, flavor, sweetness, sourness, and overall acceptability was performed. Hedonic response was judged in Sensory Evaluation Laboratory of Institute of Home and Food Sciences, Govt College University, Faisalabad.

## 3 RESULT AND DISCUSSION

### 3.1 Proximate analysis

Proximate analysis such as moisture content, ash, protein content, crude fiber, fat and NFE of milk thistle seeds grown in three different cities of Pakistan were carried out through AACC methods (2000). Table 1 revealed that in case of location, Islamabad contained highest amount of Protein, ash, moisture, and fiber that were 30.09 ± 1.50%, 2.37 ± 0.14%, 6.27 ± 0.37%, and 7.4 ± 0.37% than other cities. Whereas, in case of variety, blue variety contains higher amount than white. The findings are in harmony with the earlier work of Khan et al., (2007) who investigated the moisture, ash, fat, fiber, and protein content of milk thistle seeds as 4.24%–4.72%, 1.93%, 26.05%, 5.48%, and 26.01%. However, Malekzadeh et al., (2011) reported very low moisture content in comparison with the current results, due to climate changes and milk thistle cultivated from sandy land. Later, milk thistle crude fiber contents in the present research are in high conformity with the work of Mahmoud et al., (2015) and Jadayil et al., (1999). Furthermore, Khalil (2008) quantified low (1.5%) fiber content respectively. The finding of Mahmoud et al., (2015) are in accordance with the present observations regarding milk thistle seeds fat content, they expounded in the range of 29.68%–28.53% in two varieties. Wichtl and Bisset (1994) outlined that fat content of milk thistle was 20%–30%. Likewise, Perez et al., (2007) explained that the value of oil content of Asteraceae family is 25%. However, Khalil (2008) reported lowest 0.7% ash content in comparison with the current results, whereas Mahmoud et al., (2015) observed ash content in rang of 04.50%–03.25% in two different varieties.

**Table 1:** Mean values (%) of proximate analysis in different milk thistle varieties as well as locations

Locations	Varieties	Proteins	Ash	Fat	Fiber	Moisture	NFE
Islamabad	Blue	30.09 ± 1.50	2.37 ± 0.14	19.74 ± 0.59	7.4 ± 0.37	6.27 ± 0.37	34.13 ± 1.71
	White	27.60 ± 1.38	2.10 ± 0.08	20.79 ± 0.83	7.0 ± 0.35	6.90 ± 0.35	35.61 ± 1.78
Faisalabad	Blue	25.65 ± 1.28	2.07 ± 0.13	21.51 ± 1.29	6.40 ± 0.25	5.13 ± 0.25	39.24 ± 1.96
	White	23.01 ± 1.15	1.83 ± 0.05	22.73 ± 1.13	5.60 ± 0.33	5.60 ± 0.28	41.23 ± 2.15
Jhang	Blue	21.45 ± 1.07	1.98 ± 0.09	22.90 ± 1.15	4.73 ± 0.23	4.87 ± 0.19	44.07 ± 2.20
	White	20.74 ± 0.62	1.25 ± 0.06	23.19 ± 1.16	4.39 ± 0.13	5.01 ± 0.25	45.42 ± 2.36

### 3.2 Extraction yield

The extract yield of milk thistle seeds by soxhlet extraction ranged from 3.10 ± 0.15–6.69 ± 0.33%. In case of variety, the highest (6.69%) yield was found in **Blue** while the lowest (3.10) was found in **White**. Meanwhile, maximum (6.69%) was found in Islamabad and minimum (3.10%) was found in Jhang in case of location. Whereas it is clearly depicted from the results (Table 2) that extract yield of milk thistle seeds in microwave‐assisted extraction varied from 9.99 ± 0.49 to 6.67 ± 0.34%. The silymarin yield of milk thistle in the present research is in close conformity with the work of Jahan et al. (2016) who examined silymarin yield 6.7% in Soxhlet and 9.2%–11.2% in MAE. However, Wianowska and Wisniewski (2014) reported 8.14% yield by soxhlet extraction in comparison with the current results whereas, Subramaniam et al. (2007) observed silymarin yield 18.28 mg/g by MAE.

**Table 2:** Mean Values for silymarin quantification (mg/g) by MAE and soxhlet method in different M.T varieties as well as locations

Locations	Varieties	MAE	Soxhlet
Islamabad	Blue	1,840.6 ± 0.51	1669.5 ± 1.05
	White	1812.3 ± 1.30	1653.7 ± 1.71
Faisalabad	Blue	1804.9 ± 1.18	1644.9 ± 1.74
	White	1798.4 ± 1.27	1634.2 ± 1.14
Jhang	Blue	1792.9 ± 1.61	1624.7 ± 0.75
	White	1765.9 ± 1.50	1607.6 ± 0.99

### 3.3 Quantification of silymarin

The silymarin content of milk thistle seeds by soxhlet extraction ranged from 1669.47–1609.23 mg/g and by MAE ranged from 1,840.0–1765.08 (Table 2). Jahan et al., (2016) quantified 1656.5 mg/g silymarin content by soxhlet and 1813.3 mg/g silymarin content by MAE in milk thistle seed are in close conformity with the present research. Whereas, in comparison with current research Hammouda et al., (2014) quantified silymarin 63.1% by soxhlet. Moreover, Radjabian et al. (2008) quantified silymarin yield in the range of 23.98%–45.46% by MAE.

### 3.4 Antioxidant analysis of extract

Antioxidant activity of milk thistle seed was assessed by measuring total phenolic, flavonoid, DPPH, and FRAP. Table 3 showed that milk thistle contained total phenolics (24.17 ± 1.20–35.07 ± 1.75 mg GAE/g), total flavonoids (16.01 ± 0.80–29.09 ± 1.45 mg QE/g), DPPH (18.9 ± 0.56–25.01 ± 1.25%), and FRAP (9.73 ± 0.29–17.69 ± 0.88AAE mg/g edw). In case of location, Islamabad showed higher amount than other two cities whereas, in case of variety, blue variety showed higher results than the white variety. Earlier, Ismaili et al., (2016) yielded the flavonoid content as (33.23 mg GAE/g edw). Present results concerning total flavonoid content of milk thistle seeds are in harmony with the work of the Pereira et al. (2014) value as (20.92 mg/g). Moreover, Serce et al., (2016) finding are supported current results that milk thistle contained phenolic contents as 620.0 µg/g in ethanol extract. The finding of Pereira et al., (2014) are synchronized 23.26 mg/g with the current results. Akhtar et al., (2015) they reported total phenolic content as 20.2–85.6 mg GAE/g in methanol extract. Later, Tupe et al., (2013) investigated the low conformity of phenolic content then the present study. Earlier, Akhtar et al., (2015) investigated 20.1%–25.9% DPPH free radical scavenging activity in milk thistle in methanol and water, respectively. Later, milk thistle DPPH in the present research are in conformity with the work of Tupe et al., (2013). Furthermore, Ismaili et al. (2016) quantified the value as 353.89 mg TE/g edw, respectively. Furthermore, Ismaili et al. (2016) quantified 8.38 AAE/g edw the value of FRAP, respectively. Later, FRAP results in the present research are in conformity with the work of Serce et al., (2016) & Tupe et al., (2013).

**Table 3:** Mean Values for antioxidant activity in extract of different M.T varieties as well as locations

Locations	Varieties	TPC	TFC	DPPH	FRAP
Islamabad	Blue	35.07 ± 1.75	29.09 ± 1.45	25.01 ± 1.25	17.69 ± 0.88
	White	32.60 ± 1.63	27.12 ± 1.35	24.93 ± 1.49	16.01 ± 0.80
Faisalabad	Blue	30.09 ± 1.50	22.09 ± 1.10	23.10 ± 1.15	15.03 ± 0.75
	White	28.65 ± 1.43	20.15 ± 1.00	22.01 ± 1.10	13.93 ± 0.55
Jhang	Blue	26.90 ± 1.34	17.61 ± 0.88	20.53 ± 0.82	11.90 ± 0.36
	White	24.17 ± 1.20	16.01 ± 0.80	18.9 ± 0.56	9.73 ± 0.29

### 3.5 Antioxidant analysis of tea

Antioxidant activity of milk thistle tea was assessed by measuring total phenolic, flavonoid, DPPH, and FRAP. Table 4 showed that milk thistle tea comprised of total phenolics (15.08 ± 0.47–25.13 ± 1.50 mg GAE/g), total flavonoids (8.1 ± 0.24–15.19 ± 0.75 mg QE/g), DPPH (15.09 ± 0.75–22.08 ± 1.37%), and FRAP (7.02 ± 0.22–13.53 ± 0.81AAE mg/g edw). In case of location, Islamabad showed higher amount than other two cities whereas in case of variety, blue variety showed higher results than the white variety. Earlier, Gramza et al., (2006) yielded the phenolic contents of green tea as 20.52 g/100 g. However, Soysal (2009) reported lowest 11.52% phenolic contents in green tea than the TPC contents of current results of milk thistle tea, whereas Asghar and Masood, (2008) observed high TPC content in green tea than milk thistle tea. Furthermore, Mohammed et al., (2016) quantified 17.7–78.8 value of total flavonoid contents in different green tea brands, respectively. Kodama et al., (2010) indicate low flavonoid contents in green tea than milk thistle tea. Bhagwat et al., (2003) investigate 2.19 to 73.44 mg QE/g flavonoid contents in black tea whereas, 16.72 to 88.32 mg QE/g in different green tea brands their results revealed high flavonoid contents than milk thistle tea. Mohammed et al., (2016) revealed higher DPPH contents in green tea than milk thistle tea. Moreover, Kodama et al., (2010) finding are corroborated with the current DPPH results of milk thistle tea. Iris et al., (1999) revealed higher FRAP value in green tea, black and oolong tea than milk thistle tea. Moreover, Mohammed et al., (2016) finding are corroborated with the current FRAP results of milk thistle tea.

**Table 4:** Mean Values for antioxidant activity of tea in different M.T varieties as well as locations

Locations	Varieties	TPC	TFC	DPPH	FRAP
Islamabad	Blue	25.13 ± 1.50	15.19 ± 0.75	22.08 ± 1.37	13.53 ± 0.81
	White	23.93 ± 0.95	14.01 ± 0.70	21.47 ± 1.07	11.56 ± 0.57
Faisalabad	Blue	20.83 ± 1.04	12.23 ± 0.61	19.71 ± 0.98	9.08 ± 0.45
	White	18.53 ± 0.55	11.27 ± 0.67	18.99 ± 0.94	8.90 ± 0.44
Jhang	Blue	17.63 ± 0.70	9.37 ± 0.37	16.79 ± 0.83	8.10 ± 0.40
	White	15.08 ± 0.47	8.1 ± 0.24	15.09 ± 0.75	7.02 ± 0.22

### 3.6 Sensory evaluation

Table 5 indicated the score of different attributes of sensory evaluation. The results of present research elucidated that in case of location, Islamabad showed higher scores for color (8.66 ± 0.43), flavor (7.09 ± 0.35), sweetness (7.9 ± 0.39), and overall acceptability (8.7 ± 0.43) than the other two locations; however, in case of variety, blue shows higher score than white variety (Table 6).

**Table 5:** Mean Value for sensory evaluation of tea in different M.T varieties as well as locations

Locations	Varieties	Color	sweetness	sourness	Flavor	Overall acceptability
Islamabad	Blue	8.66 ± 0.43	7.9 ± 0.39	0.6 ± 0.01	7.09 ± 0.35	8.7 ± 0.43
	White	8.01 ± 0.40	7.2 ± 0.43	0.9 ± 0.05	7.04 ± 0.44	8.2 ± 0.41
Faisalabad	Blue	7.81 ± 0.39	6.8 ± 0.34	1.0 ± 0.04	7.00 ± 0.35	7.8 ± 0.46
	White	6.71 ± 0.34	6.6 ± 0.33	1.2 ± 0.06	6.91 ± 0.34	6.6 ± 0.33
Jhang	Blue	6.08 ± 0.30	6.4 ± 0.25	1.4 ± 0.32	6.00 ± 0.08	6.2 ± 0.24
	White	6.00 ± 0.3	6.01 ± 0.30	1.6 ± 0.09	5.06 ± 0.16	6.0 ± 0.18

**Table 6:** Mean Value for extraction yield of different M.T varieties as well as locations by MAE and Soxhlet method

Locations	Varieties	MAE	Soxhlet
Islamabad	Blue	9.99 ± 0.49	6.69 ± 0.33
	White	9.12 ± 0.46	6.50 ± 0.39
Faisalabad	Blue	8.01 ± 0.40	5.85 ± 0.29
	White	7.80 ± 0.39	5.40 ± 0.27
Jhang	Blue	7.01 ± 0.35	5.01 ± 0.25
	White	6.67 ± 0.34	4.80 ± 0.24

## 4 CONCLUSION

Nutritional profile of Blue variety is better than White whereas, in case of location, the nutritional profile of AARI is better than UAF. Blue variety holds higher antioxidant potential alongside phenolic acids and flavonoid content as compared to white. Moreover, milk thistle proved to be beneficial to cope with liver diseases and showed hepatoprotective response due to their strong antioxidant potential and presence of higher silymarin contents. In addition, milk thistle tea showed good hedonic response. Conclusively, the major clinical utility of milk thistle in diseased conditions is due to presence of biological active compounds and its high content of bio flavonoids.

## CONFLICT OF INTEREST

Authors declare that they have no conflict of interest.

## ETHICAL APPROVAL

This article does not contain any studies with human participants or animals performed by any of the authors.

## INFORMED CONSENT

For this type of study, formal consent is not required.

## Data Availability

The data that support the findings of this study are available on request from the corresponding author. The data are not publicly available due to privacy or ethical restrictions.
